# The Analysis and Research on the Influence of Sports Industry Development on Economic Development

**DOI:** 10.1155/2022/3329174

**Published:** 2022-09-10

**Authors:** Miaomiao Li, Yongfei Shi, Bo Peng

**Affiliations:** ^1^Department of Physical Education, China University of Political Science and Law, Beijing 102249, China; ^2^Department of Management, Shanxi College of Applied Science and Technology, Taiyuan 030062, China

## Abstract

The rapid development of social economy will promote the development of sports industry and then have an impact on sports economy. By using the regression analysis method, this paper compares the influencing factors of sports industry development, aiming at exploring the influence of sports industry development on economic development and its future development trend. This paper takes 12 industries of sports industry development from January 2020 to January 2022 as research objects, compares the development of sports industry of different research objects, and determines the factors affecting sports industry. We compare the promotion of different factors to sports economy and provide support for the formulation of sports industry development measures. The results show that economic growth, sports industry types, the degree of integration between sports industry and economic development, sports industry action time, and sports industry scale are the main factors affecting sports industry and promote the development of sports economy. The above indexes can improve the economic level of sports industry, and the improvement degree is about 10∼20%. Therefore, local governments and sports organizations should formulate measures to promote the economic development of sports industry from the aspects of economic growth, sports industry types, integration degree between sports industry and economic development, action time of sports industry, and scale of sports industry.

## 1. Introduction

The survey results show that the number of participants in sports industry in the world reaches 4.522 million every year, and the core number of sports industry development is 156,000, accounting for 3.45% [1]. The development of sports industry will promote the social economy, which belongs to a complex type of sports industry. It is difficult to develop sports industry. After the intervention of sports industry, it is easy to have additional effects such as economic repression and slowdown of other industries [2]. There are many ways to develop sports industry. In social economy, early industry integration and step-by-step delayed integration are the main ways. However, some scholars believe that the development of sports industry is complicated and affected by economic policies, economic strategies, economic situation, and other factors [3]. Delaying integration step by step will increase the additional impact after sports industry intervention and affect the future development trend. Some scholars have pointed out that although early industrial integration can avoid economic policies and carry out industrial integration in time, economic strategy will have an impact on economic development and reduce the accuracy of industrial development evaluation [4]. How to accurately evaluate the development of sports industry, reduce or prolong the occurrence rate of industrial inhibition, promote the industrial integration after evaluation [5], and promote the positive development trend of sports industry after intervention is the focus of research in the economic field. The research results in recent years are shown in Figure 1.

It can be seen from Figure 1 that the research on sports industry development at home and abroad is increasing day by day from 2013 to 2020, and there are more research studies on sports development under the background of big data. 80% of the studies are about the influence of sports industry development on economic development and the corresponding influencing factors. The average value fluctuation range in Figure 1 is relatively small, indicating that the development of sports industry is relatively stable. The contents in Figure 1 show that the research on the development of sports industry will become the research hotspot in the future, and the impact of industrial development on economy will be the research focus. The difficulty in the economic development of sports industry lies in the inaccurate analysis of relevant data, so it is necessary to deeply analyze the development of sports industry under big data. At the same time, under the background of big data, find out the problems existing in the economic development of sports industry and related influencing factors. Then, according to the development of sports industry, study the influence of sports industry on economic development, and do not provide the basis for the implementation of economic strategy. From the above analysis, we can see that there are significant differences in sports industry research at home and abroad. Domestic research pays too much attention to theoretical research and ignores case analysis, and foreign research results cannot be applied to China. Therefore, it is an urgent problem to strengthen the research on the influencing factors of sports industry and promote the economic development of sports industry. Therefore, from the perspective of big data, it is a hot topic to study the impact of sports industry development on economic development. On this condition, this paper finds out the influencing factors of economic development and analyzes the economic development results of two different sports industry development modes, so as to guide sports industry to play a promoting role in social economy [6]. The research on the development of sports industry in this paper mainly includes the following contents: (1) expound the development of sports industry and its impact on industrial economy under the background of big data and compare the research status at home and abroad to lead to the research content of this paper; (2) describe the development of sports industry and economic development and determine the impact of indicators for the later research content; (3) conduct comparative analysis of sports industry development and sports economic development indicators, carry out the corresponding simulation analysis, and get the research content of this paper; and (4) summarize the research content of this paper.

## 2. Research Methodology

### 2.1. Research Data and Methodology

Twelve industries in social economy from 2020 to 2022 were selected, and CPI and GDP were classified as II ∼ III. All industries were divided into research group and control group by random numbers.

The research group (*n* = 6) adopts the step-by-step delay statistical method, including 8 construction fields and 4 machinery fields, with an economic growth of 26∼59 trillion, with an average of 35.14 ± 0.13 trillion. There are 4 open developments, 8 closed developments, and 20 merged related fields. 4 are due to policy reasons, 2 are due to strategic reasons, 2 are due to market reasons, and 4 are due to other reasons. The action time was 8∼10 months, with an average time of 8.4 0.22 months. The control group (*n* = 6) used early data statistics, including 6 construction fields and 6 machinery, with an economic growth of 24∼56 trillion, with an average of 32.4 ± 0.23 trillion. There are 3 open developments, 9 closed developments, and 2 merged related fields. Two are due to policy reasons, three are due to strategic reasons, two are due to market reasons, and five are due to other reasons. The action time was from 7 to 9 months, with an average time of 8.14 ± 0.62 months. In the survey data, sports economic industries are divided into three categories, namely, intelligence industry economy, leisure industry economy and economic industry economy. Among the research data selected by the observation group, 10 items come from Class II industrial economy and 2 items come from Class III industrial economy [7].

Inclusion criteria that (1) Initial respondents; (2) Significant economic downturn, and confirmed to be economic downturn; (3) Economic restriction, inhibition, decline, and limited activities [8]; (4) Meet the requirements of post-follow-up and agree to accept post-follow-up. Exclusion criteria: (1) in a new stage of development; (2) seriously unreasonable economic structure (3) The research data comes from the official documents published by the state; (4) The industrial economic content meets the national information security requirements and does not involve internal information [9].

After collecting relevant data, the early industry integration analysis is carried out to calculate the data development of different industries. Then, the index of sports industry development is compared and analyzed, such as sports industry price, industry content, benefit, content [10], capital, and scale. Finally, use big data to find out the integration point between sports industry development and economic development and make integration analysis.

**Assumption 1 .**

The analysis of early industry integration is *Q*, the industry is *A*, the industry development index is *x*_*i*_, and the integration coefficient between industry and economic development is *w*; then, the calculation of the early integration method is shown in the following formula:

(1) $$\begin{array}{c} Q=\sum_{i}\frac{\left(w\cdot x_{i}\right)-\left(w\cdot x_{i}{}^{2}\right)}{A}. \end{array}$$

Among them, (*w* · *x*_*i*_) − (*w* · *x*_*i*_^2^) is the change value of sports industry development, *w* is the weight in the development process, and *A* is the average development value of the whole industry. Therefore, formula (1) is the role of sports industry in actual development and represents the actual situation of sports industry development.

Adopt the method of delaying integration step by step to judge the development of sports industry in the later stage, and the judgment index is the same as that of the control group. At the same time, it adopts big data analysis method, data mining, data collection, data collation, and other methods [11].

**Assumption 2 .**

The data mining background is *K*, the data mining technology is *T*, and the data collation method is *F*; then, the calculation of the step-by-step delayed fusion method *f*(*·*) is shown in the following formula:

(2) $$\begin{array}{c} f\left(x_{i},T,F\right)=\sum_{i,K}\frac{\left(w\cdot x_{i}\right)-\left(w\cdot x_{i}^{2}\right)}{A}. \end{array}$$

Among them, (*w* · *x*_*i*_) − (*w* · *x*_*i*_^2^) is the change value of sports industry development under big data, *w* is the influence weight of big data in the development process, and *A* is the average development value of the whole industry under the background of big data. Therefore, formula (2) is the role of sports industry in actual development under big data and represents the actual situation of sports industry development. Among them, formula (2) is based on formula (1), adding the background and method of big data. Because big data is a continuous variable, the continuity analysis of big data is carried out in formula (2) to improve the accuracy of result analysis.

### 2.2. Statistical Analysis

SPSS19.0 was used for normal distribution test, the measurement data were expressed by $\bar{x}\pm s$, and *t*-test was used for construction. The count data are expressed as *n* (%), and *x*^2^ chi-square test is adopted. Taking the economic development within 2 years after the intervention of sports industry as dependent variable and the indexes with significant differences between the two sports industry development methods as independent variables, the Cox ratio risk regression model was constructed to analyze the relationship between each independent index and the intervention. *p* < 0.05 represents the difference and statistical significance [12].

## 3. Research Results

### 3.1. The Comparison of Economic Development Effects of Two Analysis Methods

In terms of industry promotion time, industry integration (general integration, poor integration), economic growth (24∼35, 47∼59), sports industry type (type III), time of industry inhibition, economic development score after sports industry intervention, and negative economic effect, there are significant differences (*p* < 0.05) [13], but there are no significant differences in economic growth (36∼4), sports industry type (II type), and additional effects after sports industry intervention (*p* > 0.05). The results are shown in Table 1.

From the contents in Table 1, we can see that there is no significant difference between the indicators (*x*1∼*x*5) in the development of sports industry, so we can study the related contents. At the same time, there is no significant difference in industrial optimization time (*x*1) and industrial development intervention (*x*3). Therefore, the corresponding statistical analysis can be carried out between the study group and the control group. In addition, in the research of sports industry development level (c1∼c6), it is necessary to ensure that there is no significant difference in various economic indicators (*x*1∼*x*5). The data in Table 1 can ensure the feasibility of related research and lay a foundation for later research.

### 3.2. Single Factor Analysis of Different Economic Development within 2 Years after Sports Industry Intervention

Statistical analysis of different sports industries (S1∼S18) shows that the statistical analysis of different industries is better and can be used as analysis data for research. The results are shown in Table 2.

### 3.3. Cox Analysis Model of Influencing Multiple Factors

The indicators with significant differences in Tables 1 and 2 are taken as independent variables, and the economic development effect is taken as dependent variables, and the multi-factor Cox ratio risk analysis is carried out (see Table 3 for their respective variable assignments). The results are shown in Table 3.

It can be seen from Table 3 that there are five grades (A∼E) of factors affecting sports development, and each grade has a critical value standard set. The setting of the threshold value of each grade is mainly based on the differences of different groups in Table 2. Generally speaking, the choice of critical value is the intermediate value between two different sets of data. Cox risk analysis of the above variables shows that economic growth (*x*1), sports industry type (*x*2), integration degree between sports industry and economic development (*x*3), sports industry action time (*x*4), and sports industry scale (*x*5) are the main factors affecting the economic development effect after sports industry intervention [14], which have a significant positive impact on the economic downturn of the industry (*p* < 0.05), as shown in Table 4.

According to the data in Table 4, we can get the regression results of the impact of sports industry development on economic development, as shown in Figure 2.

As can be seen from Figure 2, scale has the most important influence on economic development, followed by time, and finally type and economic growth. It can be seen from Figure 2 that the type of sports industry, economic influence, action time, and scale of sports industry are all factors that have an impact on economic development. However, the influence of sports industry on economic development is higher than the average level. Therefore, the development of sports industry has obvious influence on economy, and its potential is huge. The main reasons for the above phenomenon are that the development of sports industry is in the primary stage of development, and economies of scale and action time are the biggest influencing factors. Therefore, under the background of big data, the impact of sports industry development on economy should be from the perspective of scale and action time.

## 4. Discussion

The rapid progress of science and technology and society increases the uncertainty of human economic development, which makes the development of sports industry have certain risks. How to better analyze the influence of sports industry development on economic development is the focus of sports industry and sports economy research at present. The influence direction of sports industry development on economic development can be divided into early industry integration and step-by-step delayed integration, and which way to choose is controversial in academic circles [15]. At present, the academic circles believe that the sports industry has an obvious impact on economic development, and the impact results can be seen within 6 months. Therefore, based on this, this paper chooses the economic data of the sports industry from December 2021 to May 2022 as the research object to analyze the impact of sports industry economy. The theoretical basis is that sports industry has less impact on economic development in 0–6 months, the early industry integration method is more accurate, and the industrial development evaluation is more ideal. However, the effect of economic development is affected by many factors, so it is necessary to find out the main factors affecting the development of economic industry, build a corresponding evaluation system, and reduce the occurrence rate of industrial inhibition [16].

The research results of this paper show that in terms of industrial promotion time, industrial development integration (general integration, poor integration), economic growth (24∼35 trillion, 47∼59 trillion), sports industry type (type III), time of industrial inhibition, economic development score after sports industry intervention, and negative economic effect, there are significant differences, but there is no significant difference in economic growth (36∼4 trillion), sports industry type (type II), and additional impact after sports industry intervention. Different analysis methods should be adopted for different economic scales, so as to improve the accuracy of analysis results. According to the complexity and economic scale of sports industry, 36 ~ 40 trillion/year is classified as medium scale, and 40 ~ 45 trillion/year is classified as large scale. Among them, the medium-sized sports industry can adopt simple evaluation methods, and the large-scale sports industry can adopt comprehensive scoring methods [17]. The scale of 47–59 trillion is larger, and the step-by-step and delayed evaluation is more accurate, which can reduce the uncertainty factors in economic development. Therefore, this method is better for the evaluation of economic development after intervention. Some scholars analyzed 102 sports industries, and the results showed that the choice of improving the development mode of sports industry needs to refer to the economic growth of the industry, and the analysis time has little impact on the analysis results, which is consistent with the research results of this paper [18]. Some scholars have proposed that the economic scale of 20–30 trillion should be integrated by early assessment and step-by-step extension.

The effect of step-by-step deferred evaluation in dealing with type III industry is better than that of early industry integration, which suggests that the sports industry of type III industry is fully developed. Although influenced by policies and strategies, the step-by-step deferred evaluation first analyzes the basic data [19] and then makes a secondary evaluation of the industrial development. Type II is only a simple analysis of industrial development and scale, which requires industrial development evaluation. The former is less affected by policies and strategies, while the latter is greater. Studies have shown that type III industries promote economic development for a long time, and the evaluation is more complicated. It is suggested to extend the evaluation time of sports industry development. Some scholars also suggested that type III industry should adopt a phased development mode of sports industry to reduce the difficulty of analyzing the development of sports industry, which is consistent with the research results of this paper [20]. The two analysis methods are relatively mature, and the focus of the economic impact of sports industry development is the evaluation of industrial development, so there is no significant difference between the research group and the control group [21].

There is no significant difference between the study group and the control group in the time of sports industry affecting economy within 1 ~ 6 months after intervention, but there is significant difference between 6 ~ 12 months and 12 ~ 18 months, and the effect of 12 ~ 18 months is significantly higher than that of 6 ~ 12 months. It is proposed to postpone the development of sports industry step by step, adjust the development of sports industry, correct the growth direction of new bones, make the industrial development tend to be evaluated in depth, and prolong the emergence time of industrial inhibition. Some research results show that economic cross-sectional evaluation is the key to the development of sports industry, and it is also the difference from other analysis methods [22]. Some scholars have studied 65 sports industries, and the results show that there is a significant correlation between the degree of industrial inhibition and bad intervention, which is consistent with the results of this study [23]. There is no significant difference between the two groups in the time from January to June. Both analysis methods are effective in comprehensive analysis of sports industry development, but there are differences in economic development scores from 1 to 12 weeks. The reason is that the analysis of the surrounding industries in the early industry analysis is not in place, and the analysis of the surrounding industries in the step-by-step delay analysis is more comprehensive [24].

Taking the indicators with significant differences in Tables 1 and 2 as independent variables and the effect of economic development as dependent variables, this paper makes a multi-factor Cox ratio risk analysis. The results show that economic growth, sports industry type, integration of sports industry and economic development, action time of sports industry, and scale of sports industry are the main factors affecting the economic development effect after sports industry intervention, which have a significant positive impact on the economic downturn of the industry.

## 5. Conclusion

Under the background of big data, the development of sports industry has certain advantages and disadvantages. Moreover, the development of sports industry will promote sports economy. How to deeply study the influence of sports production on sports economy has become an urgent problem to be solved at present. Under this background, this paper makes an in-depth analysis of the impact of sports industry development on economic development and makes an in-depth analysis in combination with the background of big data. The results show that under the background of big data, the development speed of sports industry is increasing day by day, and the promotion of sports industry to economy has been significantly improved. Among them, economic growth, sports industry types, the degree of integration between sports industry and economic development, sports industry action time, and sports industry scale are the main factors of sports industry development and promote economic development. This paper also has some limitations, mainly as follows: (1) the sports industry economic data are not enough; 2) sports industry economic data contain a large number of unstructured data. In order to simplify the data, irrelevant data or non-characteristic data are proposed, which affect the comprehensiveness of the data. Therefore, the analysis of the main factors of sports industry can provide data support and theoretical guidance for economic development. However, there are still some problems in this study, which are mainly reflected in the weight of influencing factors in the development of sports industry, as well as the time and effect of each factor on the economy. In the future research, we will focus on the analysis of the above problems and improve the research results of this paper.

## Figures and Tables

**Figure 1:** Research literature on the development of sports industry from 2013 to 2020.

**Figure 2:** The regression analysis results of sports industry development and economic development.

**Table 1:** Comparison of pathological characteristics between the two groups.

No.	c1	c2	c3	c4	c5	c6	…	*x*1	*x*2	*x*3	*x*4	*x*5
1	1	1	1	1	1	1	…	2.7500	2.5000	1.7500	2.7500	0
2	1	1	1	−1	1	−1	…	2.7500	2.5000	1.7500	2.2500	0
3	1	1	−1	1	−1	1	…	2.7500	2.5000	1.2500	2.7500	0
4	1	1	−1	−1	−1	−1	…	2.7500	2.5000	1.2500	2.2500	0
5	1	−1	1	1	−1	−1	…	2.7500	1.5000	1.7500	2.7500	0
6	1	−1	1	−1	−1	1	…	2.7500	1.5000	1.7500	2.2500	0
7	1	−1	−1	1	1	−1	…	2.7500	1.5000	1.2500	2.7500	0
8	1	−1	−1	−1	1	1	…	2.7500	1.5000	1.2500	2.2500	0
9	−1	1	1	1	−1	−1	…	2.2500	2.5000	1.7500	2.7500	0
10	−1	1	1	−1	−1	1	…	2.2500	2.5000	1.7500	2.2500	0
11	−1	1	−1	1	1	−1	…	2.2500	2.5000	1.2500	2.7500	0
12	−1	1	−1	−1	1	1	…	2.2500	2.5000	1.2500	2.2500	0
13	−1	−1	1	1	1	1	…	2.2500	1.5000	1.7500	2.7500	0
14	−1	−1	1	−1	1	−1	…	2.2500	1.5000	1.7500	2.2500	0
15	−1	−1	−1	1	−1	1	…	2.2500	1.5000	1.2500	2.7500	0
16	−1	−1	−1	−1	−1	−1	…	2.2500	1.5000	1.2500	2.2500	0
17	−2	0	0	0	0	0	…	2	2	1.5000	2.5000	0

*Note*. *x*1∼*x*5 represent the development index of sports industry, and c1∼c6 represent the economic development index.

**Table 2:** The single factors of economic development in two years after the intervention of sports industry.

The function process of industrial economy	Number of samples	Mean value	Standard deviation	Standard error	95% confidence interval	
S1	2	14.0552	0.0904	0.0640	13.2426	14.8677
S2	2	13.9648	0.3483	0.2463	10.8358	17.0937
S3	2	13.9911	0.1868	0.1321	12.3126	15.6696
S4	2	13.9941	0.2813	0.1989	11.4668	16.5214
S5	2	13.9485	0.1223	0.0865	12.8494	15.0476
S6	2	13.9556	0.0417	0.0295	13.5808	14.3304
S7	2	14.0644	0.0252	0.0178	13.8382	14.2906
S8	2	13.8775	0.0752	0.0532	13.2015	14.5535
S9	2	14.0187	0.5289	0.3740	9.2666	18.7708
S10	2	13.8306	0.3451	0.2441	10.7296	16.9315
S11	2	13.7954	0.2969	0.2100	11.1277	16.4630
S12	2	14.1974	0.1119	0.0791	13.1923	15.2025
S13	2	13.9596	0.0293	0.0207	13.6966	14.2226
S14	2	13.9339	0.1121	0.0793	12.9263	14.9415
S15	2	14.0720	0.0612	0.0433	13.5218	14.6222
S16	2	13.7139	0.4219	0.2983	9.9236	17.5042
S17	2	14.3579	0.1048	0.0741	13.4164	15.2994
S18	2	14.1618	0.1232	0.0871	13.0551	15.2685

*Note*. S1∼S18 represent the action process of sports industry development on economic development.

**Table 3:** Impact grade analysis.

Development of sports industry		Fusion	Economic development	
A	C	D	E	B
D	A	B	C	E
E	B	C	D	A
C	E	A	B	D
B	D	E	A	C

*Note*. A∼E represent different grades, and grade A is the lowest.

**Table 4:** Risk analysis results of multi-factor Cox ratio.

Number of factors	Score	Degree of influence	Types of sports industry	Qs	*p*
1	85.0490	84.8770	1760.2541	0.0009	0.9999
2	83.7128	84.1403	1760.5481	0.0057	0.9999
3	84.2204	84.2383	1760.5715	0.0000	0.9999
4	84.2370	84.3283	896.2434	0.0008	0.9999
5				0.0007	0.9999

## Data Availability

The data used to support the ﬁndings of this study are available from the corresponding author upon request.
